# Designing a Predictive Model for Antiretroviral Regimen at the Antiretroviral Therapy Center in Chiro Hospital, Ethiopia

**DOI:** 10.1155/2021/1161923

**Published:** 2021-10-29

**Authors:** Gadissa Nemomsa, M. Azath

**Affiliations:** ^1^Computer Science Department, Oda Bultum University, Chiro, Ethiopia; ^2^Faculty of Computing & Software Engineering, Arba Minch University, Arba Minch, Ethiopia

## Abstract

Nowadays, the huge amount of patient's data significantly increases with respect to the time in repositories and data mining is increasingly used as an emerging research area in medical fields for extracting useful and previously unknown insights/patterns from the repository data. These unknown patterns/hidden insights can help in discovering new knowledge hidden in these data repositories. From the observation, different ARV regimens were ordered for different patients. However, combination of these drugs causes different side effects on the patients. It has been observed that there was a lack of predictive studies and designed models available in hospitals specifically ART Centers that accurately determine or classify the patient's ARV regimen to TDF + 3TC + EFV, TDF + 3TC + NVP, AZT + 3TC + ATV/R, AZT + 3TC + LPV/R, TDF + 3TC + LVP/R, TDF + 3TC + ATV/R, 8888, and ABC + 3TC + LPV/R. In order to solve these kinds of problems, we built an accurate classifier system or model using parameters like Patient Age, Patient Encounter Day, Patient Encounter Month, Patient Encounter Year, Patient Weight, Patient CD4 Count Adult, Patient TB Screen, Patient Following WHO Stage, Patient CD4 Percent Child, Patient Regimen Specify, Patient Regimen, and so on. The general objective of this research was predictive modeling for the patient's ARV regimen class through data mining techniques so as to improve them. The study used the CRIPS-DM methodology to find and interpret patterns in repositories. A decision tree (J48 and Random Forest) algorithm was used for classification. Using all tested classifiers, the investigation of the study shows that the total accuracy was more than 60%. On the other hand, among different classifications, class H (ABC + 3TC + LPV/R) has shown the worst prediction. But it was revealed that the J48 classifier relatively produces higher classification accuracy for the D (AZT-3TC-NVP) regimen. Here, classification depended on the selected parameters, which revealed that prediction accuracy value differed among all classifiers and the selected attributes. Finally, the study concluded that data mining can be used as a significant technique to discover patient regimen based on salient affecting factors with 96.1% precision achieved. Ensemble learning resolves the categorizing models of greater anticipating performance with different learning algorithms. This model aligned with sentimental investigation to magnify the appearances of the dataset either from the social media or from primary data collection. The empirical investigation with different parameters shows the detailed improvement of their learning methods.

## 1. Introduction

Ethiopia has nearly 800,000 HIV patients, and the total population prevalence is about 1.5%. However, as different investigation shows, the transmission annually increases, and the situation is become worst and approximately 1.3 million patients living with the virus, especially adults, are highly affected in the country [1].

Ethiopia is among the least developing countries facing high infectious, injuries, and problems including HIV. As a matter of fact, the country has the Antiretroviral Treatment (ART) Center to protect lives, also to reinstate the mental utilities to improve, and to encourage the morality of patients [2]. Different report indicates the population of HIV positive registered to ART annually increasing. Even though the reports indicate growing number of HIV patients, the center could not get analyzed prediction model as per parameter obtained from ART database [3].

An ARV regimen is mixed or grouped HIV drugs or medicines, which is used to treat HIV patients such that antiretroviral therapy (ART) uses HIV medicine to treat the infection. Patients on ART daily take a mixed or combined HIV drugs or medicines, which are ARV regimen [1, 2].

In general, the combination of HIV regimen includes or mixed three HIV medicines from at least two different drug combination classes, and this selection of HIV medicine/drug depends on a person's individual needs. Although the drug taken from ART Center alone could not cure patients, but they should eat more, control weight, and feel good, and their bodies are more robust to recover and fight against infections. As patients are well cared for, they care for their family and become of more benefit to society and economy of the country [1]. The virus has affected the lives of millions and has left many orphans. Ethiopian government took several footsteps in declining further virus spread and encouraging treatment demand for patient care and support for HIV patients [4]. Before 1996, being HIV positive was nearly equal to death, but later with the investigation of collective antiretroviral handling, HIV/AIDS is shifted from death sentence to chronic controllable disease [2].

Data mining is the extensive extraction of hidden data and possibly getting meaningful information from huge data sources [5]. The exploration is not only discovering but also the procedure of data analysis from different views of parameters to achieve new patterns. Hence, the process of data mining passes through the following basic elements: preprocessing, transformation, and loading the clean data in systems/tools [4]. It also manages easily the source of data using different ways of database system and is able to extract data accessible to domain expert. So data mining techniques can analyze the data using application software and viewing extracted pattern [2]. The main benefit of this study was to investigate designing and modeling ARV regimen and also determining and predicting the patient's antiretroviral regimen on ART Center, which determines and categorizes the patient's antiretroviral regimen in to classes like TDF + 3TC + EFV, TDF + 3TC + NVP, AZT + 3TC + ATV/R, AZT + 3TC + LPV/R, TDF + 3TC + LVP/R, TDF + 3TC + ATV/R, and ABC + 3TC + LPV/R based on obtained variables [6]. Remarkably, data mining is solving problems through analyzing data, which is already present in huge quantities in order to discover unknown patterns and rules [4]. It has been observed that many problems are considered while choosing ARV regimen, and choosing HIV medicine/drug depends on a person's individual needs [7]. So the healthcare provider follows the following factors: patients that may be living with other different diseases, such as heart diseases, way of transmission, pregnancy, side effects of drug itself, the potential compatibility of the medicine with HIV patients, and getting convenience toward taking regime [8]. Different ARV regimens are ordered for different patients. However, combination of these drugs have different side effects on the patients. So parameters like Patient Age, Patient Encounter Day, Patient Encounter Month, Patient Encounter Year, Patient Weight, Patient CD4 Count Adult, Patient TB Screen, Patient Following WHO Stage, Patient CD4 Percent Child, Patient Regimen Specify, Patient Regimen, and so on have great impact on patient living with HIV/AIDS. In ART Center, manually ordering ARV regimen by itself has a problem and is more sensitive to error. So the disordering of the regimen without considering the aforementioned parameters could cause great side effects on patient side. From deep review, the exploration and application of data mining techniques for designing predictive models are not yet fully exploited to support antiretroviral therapy for minimizing the risk of HIV patients. This problem creates thrust to explore and analyze the potential applicability of data mining techniques in designing a predictive model that can predict ARV regimen based on patients' previously stored data and discover deployed patterns that could identify the most determinant factors on patients' ARV regimen.

In many organizations, plenty of data have been described as data-rich but information-poor society/institute. Today, in this world, big amounts of data are collected daily so that it is very necessary to investigate and extract hidden use of full knowledge from such huge data. Data mining is one of the best procedures of investigating meaningful and new knowledge from a vast amount of data sources. These data sources can involve different sources like databases, the web, data warehouses, and data repositories [4]. It is an interdisciplinary domain and has more alternative possibility named, which is knowledge mining from data.

Data mining considered as a CRISP process model is an industry standard process including the series of procedures that are frequently included in a data mining domain [9]. CRISP-DM offers a uniform context (framework) for experience documentation, and it is used and applied broadly in various industries with different types of data. It naturally includes cleaning data, selection of data, integration, transformation, pattern detection, pattern analysis and evaluation, and deployment [5].

## 2. Literature Review

The research study [10] states that in the context of India, as the preponderance of fidelity to antiretroviral therapy, it is considered as the world's largest pandemic. In India, women are more affected than men. The impacts of the patients are addressed to depression and stress. The government is concentrating on the infected people by allocating more budget through Ministry of Health and Family.

The study from Pakistan [11] on the antiretroviral therapy was influenced by humans who were infected with HIV, which seriously affected their immune system. If the drug was not given properly to those victims, they will be at risk of more infections. A nonlinear control algorithm approach was used to control the readiness of the HIV patients. Their system was aligned with more backstepping controls to check and improve the efficiency of the drug to the infected persons on their T cells.

The study in [12] postures the South African ambience of infected patients who suffered with different problems like drug resistance, stress, and stigma. Their research helps the community level feasibility to point out the problems of the patients. A study [13] from Sub-Saharan Africa states that they follow up adherence to treat the HIV patients. They distinguished adherence and nonadherence patients' clinical data, which addressed the nonadherence of patients facing more problems like failure of immune systems and fatigues. The results show around 72.9% of adherence patients are saved and reduced the transmissions from HIV + mother to child, while [14] Sub-Saharan Project 2030 results, through their simulation model, suggest that antiretroviral drugs reduce the rate of HIV victims, especially in case of adults. In the study conducted in Zambia [15], nearly 1.9 million people are affected by HIV. The researchers proposed ART helps the HIV infected patients of long-term survival, and they suggest the government to allocate the budget to sustain this technique in forthcoming days. A study [16] was conducted in 2021 to treat the HIV patients with a new care service as LTFU (lost to follow-up). The LTFU service was very helpful among the adults living in Sub-Saharan area. Meta-analysis of LTFU achieved greater benefits for the patients who are suffering from HIV. A collaborative study from Malawi, South Africa, and Zambia [17], which addressed the mortality rates, is increasing in these countries. Viral load (VL), CD4 count, and different monitoring mechanisms had shown the results of mortality due to several factors. They implement stochastic simulation model to learn the effects of VL monitoring on mortality rate. The usage of VL with ART reduces the rate of mortalities, and the patient's immune system was also better.

A study [18] from Southeast Coast of Africa shows they faced tremendous difficulties to treat the HIV victims to follow up their health. There was a high level of possibility to transmit the disease from mother to child. The patient's data was monitored for mitigating these risks, with different levels of prevention measures taken to reduce those problems. Fidelity of victims faced numerous problems like increasing number of HIV patients and even pediatric cases were increased. To eradicate the above stated risk, they launched different control mechanisms such as SMS reminders and mobile health applications that are used to notify the HIV + mothers to prevent themselves. With these mechanisms, the number of cases is reduced and many children are saved from this pandemic.

The study in [19] states that the different parameters were used to predict different HIV-1 victim's clinical data with sexually transmitted infections (STI); from that they focus their attention toward confidence to increase the patients' health. Their estimated clinical data focused on the capability of increasing the immune system of the victims.

In a study conducted in the USA [20], HIV-1 infection dynamic model was designed and evaluated with their data to ease the improvement in human beings. Bootstrapping is used in order to correlate the different parameters. Among those parameters, confidence is considered more crucial to interpret their clinical proofs, though this efficacy of the immune system was much improved. In a study from USA [21], the researchers proposed CART (Combination Antiretroviral Therapy) as a mixed ART drug, which was given to the HIV + patients through blood plasma technique. With this usage, the level of mortality was decreased.

A study in the Middle East [22] reveals that refugee crisis leads to the increasing cases of HIV, tuberculosis, and malaria. To eradicate these challenges, the Global Fund has taken many initiatives to fight again these cases. There is a lack of health infrastructure due to their internal conflicts. By 2030, the Global Fund commitment is planning to save millions of refugees who are facing these kinds of diseases. Awareness programs are given to people to maintain their safety.

According to the study conducted in Ethiopia [23], people who are surviving with HIV are adherent with antiretroviral therapy. Almost 81% of them are infected through unprotected sexual intercourses; the researchers recommended to go ahead with adherence to reduce the HIV victims. This helps the patients under treatment to increase their immune insufficiency. The study in [24] stated that according to the WHO survey in 2018 and 2019, nearly 36 million people are infected around the world with human immunodeficiency virus (HIV). The rates of mortality are increasing due to poor adherence. The researchers are showing in their results that Tigray, Ethiopia, was heavily populated with this disease; also, they recommend creating awareness to rural part of Ethiopia to increase the drug adherence of ART. A study in [25] presenting the viability usage of data mining with ART toward the HIV positive victims shows the greater performances with prediction rate of 80.5%, while [26] designed ART predictive model achieving their results of 66% with different hospital data in Amhara Region, Ethiopia. Knowledge Discovery in Databases (KDD) model is used to maintain the HIV + patient's details.

Investigation of [27] by sentiment analysis, also called opinion mining, describes the NLP (Natural Language Processing), which shows the perception of the text. This sentiment analysis extracts knowledge from different sources. The investigation with ensemble shows the aggregation model for making effective automation to filter different distribution. The results with different algorithms indicate the accuracy level of 94.7% to strengthen their findings.

The study in [28] addresses the elimination of social media text documents while eradicating the information from the datasets. The cutback data are identified and classified into databases to retrieve them in the future to yield the effectiveness. The researchers implement two ways of pruning for finding the missing values in their datasets. They achieved the better performances by using the method of ensemble pruning to build the efficient sentimental and confidential messages.

The study in [29] represents that online media platforms show the nonnatural symbolic language included with sarcasm. Symbolic languages are the rudiment of sentiment analysis. Humorous text comes under the symbolic language, which identifies the sarcasm dataset from the social media. Different data mining algorithms are used to analyze the ensemble methods to predict the better accuracy results.

Experimentation in [30] states that the usage of sentiment analysis differentiates the obtained text into real and imaginary. Even sentiment analysis may elicit the information's from nonstructured text values to judge based on the preferences of different inputs. This study confesses the involvement of students to be very efficient and assessed. The researchers applied around 700 students' details notified in Turkish language. The results are very much satisfied for evaluating this algorithmic approach.

The study in [31] confesses that the recognition of sarcasm is a hard task in NLP due to preponderance of social platforms. The researchers applied deep neural networks and language models for the text criticizing messages from social media data. They designed three-layer frameworks to pinpoint the criticizing text messages to obtain the exact outputs. They achieved the accurate output efficiency of 95.30% for false/criticizing messages from the social media data.

### 2.1. Overview of Data Mining and CRISP-DM Predictive Model

Predictive model performs insinuation on the present recorded data to predict how new information will be extracted and describe the characteristics of a dataset [2]. Classification is required for the model because it is more understandable by humans, it is highly accurate and interpretable, and it quickly build huge training database [5]. The training data are shown by labels that denote the class of the observations and classifying the new dataset on the training set. Classification models predict categorical class labels and predict continuous valued using prediction models [2, 5]. Hence, in this study, the training data was classified using classification approach.

### 2.2. Decision Tree

Decision tree is one of the data mining techniques and flow-chart-like tree structure and is used to build classification models [5]. It is one of the predictive modeling methods which can be used in data mining, statistics, and machine learning. The trained data path from root to the leaf precedes the best satisfied rule as per the labeled class. A decision tree is one of selected algorithms, which can be directly transformed to rule induction algorithms that can be used as the best popular technique in procedure of knowledge representation because of its easiness and unambiguousness [1].

Based on the critical review of domain specific and focused research studies cited above, researchers observed a crystal clear research gap in terms of accuracy of results, technique used, designing model, and parameters consideration that typically influence the patient's ARV regimen. Hence, the research results significantly revealed new ideas and new knowledge contribution and provided a solution toward ordering and identifying extensively extracted patterns or ARV regimen for patients in vibrant way to the expert/ART Center.

### 2.3. Summary of the Literature

ART model is recommended to be used for the patients who are suffering from HIV. Viral load (VL) helps to reduce the death rate of people who are infected with HIV. Adherence should follow up the patients in order to eradicate the problems and increase the patient's immune systems. In the coming years, for example, by 2030, we should join the Global Fund Commitment to reduce the mortality rate of AIDS patients. KDD models are witnessed to have the data about those victims who are suffering from HIV. Ensemble learning resolves the categorizing models of greater anticipating performance with different learning algorithms. This model aligned with sentimental investigation to magnify the appearances of the dataset either from the social media or from primary data collection. The empirical investigation with different parameters shows the detailed improvement of their learning methods.

## 3. Research Design and Methodology

The research is based on the CRIPS-DM modeling technique. In order to achieve the desired goal of the research, the study followed CRIPS-DM process model. As the concepts of the CRISP-DM process model, the steps of a knowledge or pattern extracting process involve six phases [32].  Figure 1 represents the methodology of the research.

### 3.1. Identifying Problem and Business Understanding

In this study, identifying and understanding the problem was the initial journey of the work. After understanding the problem to be briefly addressed, the next step was understanding and identifying available data source. Understanding and identifying data source was identified by observing and interviewing the domain expert.

### 3.2. Data Collection

Primary data, which states the data, was collected initially to gather information about the domain [10]. Primary data is used to gather fresh data in the early stage [31]. The significant data was collected from patient repository data, which was in ART Center, Chiro Hospital, Ethiopia; that is, 3115 records were collected for conducting the experiment. The required parameters like Patient Age, Patient Encounter Day, Patient Encounter Month, Patient Encounter Year, Patient Weight, Patient CD4 Count Adult, Patient TB Screen, Patient Following WHO Stage, Patient CD4 Percent Child, and Patient Regimen Specify were collected from repository data. Ultimately, the structural was collected for subjective measures to evaluate the predicted model (extensively extracted new knowledge) [33].  Figure 2 represents the data collection procedure, which was followed during this research.

### 3.3. Data Preparation and Preprocessing

The orders or tasks, such as processing and cleansing, were done in order to make the data more appropriate for the specific data mining tools, which was effectively used in the study. This constitutes preprocessing data shown in Figure 3:

- Data cleaning was as follows: attempting to correct inconsistency, handling noisy data, and handling missing data fields and integrating, transforming, and preparing the processed data in a file format acceptable to the tool or software that has been implemented.
- Integration of data was as follows: the process of merging prepared data, which is obtained from different repositories by reducing and avoiding redundancies and inconsistencies to improve the accuracy
- Data transformation and selection were as follows: to transform or consolidate data into forms suitable for mining strategies like attribute construction, aggregation, and normalization. In this study, data preparation and preprocessing constructing a dataset from one or more data sources is used for exploration and modeling.

### 3.4. Data Mining Technique

In data mining, many classification techniques, such as rule based, genetic algorithms, naïve Bayes, nearest neighbor method, neural network, and decision trees, are the most used methods in data mining [5]. In this research study, to understand and generate rules to implement the handling of dimensional data, time, and accuracy, the decision tree algorithms are selected selected for classification models as data mining algorithms. DT is selected for the reason of handling irrelevant attributes through information gain, being robust against skewed distributions, and being easy to interpret (visualize and manipulate) [4]. Ultimately, after comparing the accuracy result of two selected classifiers of DT, the overall best model of algorithm was selected. Feature selection and model building were selected by modifying the values of the parameters in order to improve the patient regimen of the predicted model.

#### 3.4.1. Tool Selection

The Waikato Environment for knowledge analysis (WEKA) is a mostly used tool (software) in data mining research [32]. It is an open-source software, which can support numerous typical data mining components or tasks. To select a data mining tool, some parameters were taken into consideration, such as data mining technique, which could perform classification technique. In consideration of numerous types of data mining software, Weka 3.9 tool was selected for the research study. The tool is selected due to its open source (obtained free), being more essentially modifiable and maintainable, and being completely implemented in java and platform. It has prediction and classification features [2, 32], which are essential for the research.

## 4. Result Evaluation/Interpretation

Model results were evaluated in the perspective framework of the business purposes recognized in business understanding. Data analysis and evaluation processed the collected information and determined the conclusions, significance, and implications of the findings [34]. So, after mining the required pattern, the interpretation and evaluation of the mined patterns will be accomplished [35]. In this study, evaluation was to represent the result in an appropriate way. The performance of the algorithms adopted in the study was measured and evaluated based on their accuracy and recall and precision, and the rule was generated from the preferred model. The result was predicted and performed using the selected algorithms.

## 5. Deployment

Data mining validated previous knowledge extracted and verified unpredicted and valuable relationships [4]. Based on the new knowledge extracted, a model was obtained that could be applied to domain experts for the purpose of prediction [36].

## 6. Experimentation and Result

### 6.1. Experiment

Two of the classifiers conducted in the model building like decision tree algorithm (J48 and Random Forest) were applied on datasets with their default parameters and with new adjusted parameter values.  Table 1 summarizes the achieved results and performance of the selected classifiers using test model.

In order to compare the best model, precision, recall, and the accuracy (correctly classified instances) of the classes were used for different classifiers based on their test model. The following figure compares and contrasts each classifier based on their precision, recall, and accuracy.

From Figure 4 and Table 1, it was observed that the recall and accuracy do not have much difference in all experiments. In experiment I, both recall and accuracy values were found to be high, that is, 95.7% and 96.12%, respectively. But in both test models, they became low in experiments I and II, during percentage split of 80%. Likewise, the precision was high (96.1%) when compared with other experiments. However, the other experiment II has not much gap values when it is compared with experiment I. J48 unpruned tree model was selected with its performance that could predict patient regimen (AZT-3TC-EFV, TDF + 3TC + EFV, TDF + 3TC + NVP, AZT + 3TC + ATV/R, AZT-3TC-NVP, TDF + 3TC + LPV/R, AZT-3TC-NVPkid, and ABC + 3TC + LPV/R), that is, 96.12% accurate prediction using true positive and true negative with the absolute error (0.0105) that could also measure values of the error among actual and predicted models with kappa statistic (0.9494); hence, it was frequently 1.0, which indicates being fully covenant. Therefore, in this study, the model created using J48 unpruned tree scored better regimen and hence is selected for further analysis/rule tracing for provided dataset.

### 6.2. Performance Comparison between the Applied Classifiers

The compared results of the conducted classifiers for the experimentation (true positive rate, 10-fold cross validation) are summarized and presented in Figure 5.

The obtained result shows that the classifier J48 performs better; that is, it has the highest accuracy among the others. However, both applied classifiers were recording with total accuracy under 96.2% that means the obtained error rate was almost medium and the expected predictions were not relatively dedicated. On other hand, the total accuracy of the Random Forest classes was concerned; it was observable that the expected predictions were low for TDF + 3TC + LPV/R class and the worst for the ABC + 3TC + LPV/R class; thus, the Random Forest classifier was unconditionally less sound to predict the classes. Therefore, the more accuracy was realized for the AZT-3TC-NVPkid, followed by the AZT + 3TC + ATV/R and TDF + 3TC + NVP classes. The predictions for the AZT + 3TC + ATV/R and TDF + 3TC + NVP classes were more precise than for the other classes, and from tested classifiers, the total accuracy indicated were more than 60%. The decision tree classifier (J48) was the most reliable because it performs with the highest accuracy than the others. But as both classifiers comparatively observable, the Random Forest classifier was less accurate than the J48.

## 7. Conclusion

ART model was useful to reduce the death rate of HIV positive persons. ART model was useful to reduce the death rate of HIV positive persons. Likewise, ensemble learning model shows different learning algorithms to enhance the performance of the datasets. The researchers resolved that the experiments conducted in this research showed that patient's ARV regimen was analyzed significantly by identifying influencing factors. It is also possible to significantly use to minimize patients from risk and enhance medical care of their patient; that is, it could increase efficiency to take appropriate measures or plan to treat in early strategies.

In this research, each patient's regimen was identified as either A or B/D/C/E/F or H based on the determinant attributes. The study outcome will powerfully help the medical staff to know properly ordering antiretroviral regimen rather than giving manually different combination of ARV regimen, which would be genuine attention to reduce side effect of ARV regimen ordering. This research investigated figuring out the patient regiment from huge data in order to identify patient at risk, which is base to develop model and also to help hospital (medical staff) by early identifying patient's status to get information about patient for better planning and formulating medical policies for utilizing medical facilities in better planning. Thus, data mining techniques, particularly the decision tree (J48) technique, can be known as well, applicable to predicting patient regimen pattern. Attributes considered for patient regiment datasets in this study were Patient Age, Patient Encounter Day, Patient Encounter Month, Patient Encounter Year, Patient Weight, Patient CD4 Count Adult, Patient TB Screen, Patient Following WHO Stage, and Patient CD4 Percent Child.  Figure 6 shows the classifiers performance on different classes [10, 37–39].

## 8. Recommendation

Important parameters like diet, pregnancy (prelabor, postlabor), opportunistic infection (bacterial, fungal, viral, and parasitic), and sexual transmission infections were recommended for further study. Other data mining methods like neural network and vector machine were not considered for testing and prediction. Such parameter and method will increase the accuracy and reliability of the result.

## Figures and Tables

**Figure 1:** CRISP-DM methodology [32].

**Figure 2:** Data collection methods/techniques.

**Figure 3:** Basic flow for designing model of research work.

**Figure 4:** Comparison of conducted experiments.

**Figure 5:** Comparison of conducted experiments (using test mode).

**Figure 6:** Classifier's performance comparison on predicted classes.

**Table 1:** Summary of experimental result of classification algorithms for dataset.

Experiments	Classifiers	Test options	Precision (%)	Recall (%)	Accuracy (%)
I	J48-C 0.25-M 2	10-FCV	96.1	95.7	96.12
		PS 80%	95.4	95.3	95.3

II	Random Forest-P 100-L100	10-FCV	95.2	95.1	95.7
		PS 80%	94.6	94.4	94.3

Exp.: experiment, 10-FCV: 10-fold cross validation, and PS: percentage split 80%.

## Data Availability

This research was conducted with almost 3115 patients' data from Chiro Hospital, Ethiopia. The researchers are not ready to disclose the data in regard to the privacy policy of both patient and hospital and are not publicly available due to their restrictions.

## References

[1] Chanthaweethip W., Guha S. (2012). Temporal data mining and visualization for treatment outcome prediction in HIV patients. *Procedia Computer Science*.

[2] Cerna P. D., Jemal Abdulahi T., Abdulahi T. J. (2016). Prediction of anti-retroviral drug consumption for HIV patient in hospital pharmacy using data mining technique. *International Journal of Information Technology and Computer Science*.

[3] Awoke Ayele T., Worku A., Kebede Y., Zuma K., Kasim A., Shkedy Z. (2019). Model-based prediction of CD4 cells counts in HIV-infected adults on antiretroviral therapy in Northwest Ethiopia: a flexible mixed effects approach. *PLoS One*.

[4] Han J., Kamber Jian Pei M. (2012). *Data Mining Concepts and Techniques*.

[5] Rodriguez J., Prieto S., Correa C. (2018). Prediction of CD4+ cells counts in HIV/AIDS patients based on sets and probability theories. *Bentham Science Publishers*.

[6] Who (2017). *Dosages of Recommended Antiretroviral Drugs*.

[7] Gendelman H. E., McMillan J., Bade A. N., Edagwa B., Kevadiya B. D. (2019). The promise of long-acting antiretroviral therapies: from need to manufacture. *Trends in Microbiology*.

[8] Obed A. (2019). A predictive model for demand for first-line antiretroviral (ARV) drugs using data mining techniques. *Journal of Health & Medical Informatics*.

[9] Gebre Mariam B., Haile Mariam T. (2015). Application of data mining techniques for predicting CD4 status of patients on ART in Jimma and Bonga Hospitals, Ethiopia. *Journal of Health & Medical Informatics*.

[10] Azath M., Melese Z., Abey B. (2021). Deep learning-based image processing for cotton leaf disease and pest diagnosis. *Journal of Electrical and Computer Engineering*.

[11] Butt R. S., Ahmad I., Iftikhar R., Arsalan M. (2019). Integral backstepping and synergetic control for tracking of infected cells during early antiretroviral therapy. *IEEE Access*.

[12] Chakraborty A., Hershow R. C., Qato D. M., Stayner L., Dworkin M. S. (2020). Adherence to antiretroviral therapy among HIV patients in India: a systematic review and meta-analysis. *AIDS and Behavior*.

[13] Heestermans T., Browne J. L., Aitken S. C., Vervoort S. C., Klipstein-Grobusch K. (2016). Determinants of adherence to antiretroviral therapy among HIV-positive adults in sub-Saharan Africa: a systematic review. *BMJ Global Health*.

[14] Estill J., Ford N., Salazar-Vizcaya L. (2016). The need for second-line antiretroviral therapy in adults in sub-Saharan Africa up to 2030: a mathematical modeling study. *The Lancet HIV*.

[15] Kabaso E. M., Currie C. S. M., Brailsford S. C. Simulating the provision of antiretroviral therapy in Zambia.

[16] Kebede H. K., Mwanri L., Ward P., Gesesew H. A. (2021). Predictors of lost to follow up from antiretroviral therapy among adults in sub-Saharan Africa: a systematic review and meta-analysis. *Infectious Diseases of Poverty*.

[17] Estill J., Egger M., Johnson L. F. (2013). Monitoring of antiretroviral therapy and mortality in HIV programmes in Malawi, South Africa and Zambia: mathematical modelling study. *PLoS One*.

[18] Davey J., Nguimfack A., Hares S., Ponce W., Sousa C., Traca D. Evaluating SMS reminders in improving ART and PMTCT adherence in Mozambique: challenges in achieving scale.

[19] Banks H. T., Davidian M., Hu S., Kepler G. M., Rosenberg E. S. (2008). Modelling HIV immune response and validation with clinical data. *Journal of Biological Dynamics*.

[20] Baraldi R., Cross K., McChesney C. Uncertainty quantification for a model of HIV-1 patient response to antiretroviral therapy interruptions.

[21] Jagarapu A., Mann R., Piovoso M. J., Zurakowski R. Positive feedback through inflammation creates bistable behavior in HIV tissue sanctuaries.

[22] https://www.theglobalfund.org/media/7642/publication_middleeastresponse_focuson_en.pdf?u=636917026580000000.

[23] Ejigu M., Desalegn Z., Mulatu B., Mosisa G. (2020). Adherence to combined antiretroviral therapy and associated factors among people living with HIV attending nekemte specialized hospital, Oromia, Ethiopia: a cross-sectional study. *HIV*.

[24] Gebreagziabher T. T., Woldemariam G. T. (2020). Antiretroviral treatment adherence and determinant factors among adult people infected with human immunodeficiency virus in eastern tigray general hospitals, Northern Ethiopia, 2019. *HIV*.

[25] Chala T. D. (2019). Data mining technology enabled anti retroviral therapy (ART) for HIV positive patients in gondar university hospital, Ethiopia. *Bioinformation*.

[26] (2016). Application of data mining techniques on pre art data: the case of felege hiwot referral hospital. *International Journal of Research Studies in Computer Science and Engineering*.

[27] Onan A., Korukoğlu S. (2016). A feature selection model based on genetic rank aggregation for text sentiment classification. *Journal of Information Science*.

[28] Onan A., Korukoğlu S., Bulut H. (2017). A hybrid ensemble pruning approach based on consensus clustering and multi-objective evolutionary algorithm for sentiment classification. *Information Processing & Management*.

[29] Onan A., Tocoglu M. A. (2020). Satire identification in Turkish news articles based on ensemble of classifiers. *Turkish Journal of Electrical Engineering and Computer Sciences*.

[30] Toçoğlu M. A., Onan A. (2020). Sentiment analysis on students’ evaluation of higher educational institutions. *Advances in Intelligent Systems and Computing*.

[31] Onan A., Tocoglu M. A. (2021). A term weighted neural language model and stacked bidirectional LSTM based framework for sarcasm identification. *IEEE Access*.

[32] Teshome Yimer Y., Worku Yalew A. (2015). *Magnitude and Predictors of Anti-retroviral Treatment (ART) Failure in Private Health Facilities in Addis Ababa, Ethiopia*.

[33] Azath (2020). Statistical machine translator for English T tigrigna translation. *International Journal Of Scientific & Technology Research*.

[34] Reepalu A. (2017). *Antiretroviral Treatment at Ethiopian Health Centers*.

[35] Vilar S., Friedman C., Hripcsak G. (2017). Detection of drug-drug interactions through data mining studies using clinical sources, scientific literature and social media. *Briefings in Bioinformatics*.

[36] Olson Dr. D. L., Delen Dr. D. (2008). *Advanced Data Mining Techniques*.

[37] Rohr K., Ive P., Horsburgh R., Berhanu R. (2016). *Developing a Predictive Risk Model for First-Line Antiretroviral Therapy Failure in South Africa*.

[38] Paul R. H., Cho K. S., Belden A. C. (2020). Machine-learning classification of neurocognitive performance in children with perinatal HIV initiating de novo antiretroviral therapy. *AIDS*.

[39] Williams B. G., Lima V., Gouws E. (2011). Modelling the impact of antiretroviral therapy on the epidemic of HIV. *Current HIV Research*.

